# SegChaNet: A Novel Model for Lung Cancer Segmentation in CT Scans

**DOI:** 10.1155/2022/1139587

**Published:** 2022-05-14

**Authors:** Mehmet Akif Cifci

**Affiliations:** Dept. of Computer Engineering, Bandirma Onyedi Eylul University, Balikesir, Turkey

## Abstract

Accurate lung tumor identification is crucial for radiation treatment planning. Due to the low contrast of the lung tumor in computed tomography (CT) images, segmentation of the tumor in CT images is challenging. This paper effectively integrates the U-Net with the channel attention module (CAM) to segment the malignant lung area from the surrounding chest region. The SegChaNet method encodes CT slices of the input lung into feature maps utilizing the trail of encoders. Finally, we explicitly developed a multiscale, dense-feature extraction module to extract multiscale features from the collection of encoded feature maps. We have identified the segmentation map of the lungs by employing the decoders and compared SegChaNet with the state-of-the-art. The model has learned the dense-feature extraction in lung abnormalities, while iterative downsampling followed by iterative upsampling causes the network to remain invariant to the size of the dense abnormality. Experimental results show that the proposed method is accurate and efficient and directly provides explicit lung regions in complex circumstances without postprocessing.

## 1. Introduction

Lung cancer is the leading cause of cancer-related death globally. According to the World Health Organization (WHO) forecasts for 2019, cancer is the major or second leading cause of death in 112 of 183 nations, and it ranks third or fourth in an additional 23 countries before the age of 70 [1]. The 5-year survival rate is approximately 34% for patients with early-stage, resectable cancer, while the 5-year survival rate is less than 10% for unresectable cancer. Therefore, early identification and diagnosis of lung cancer are essential in enhancing patient treatment results. When images reveal the existence of a tumor, it is critical to histopathologically evaluate diagnostic samples collected by fiberoptic bronchoscopy following National Comprehensive Cancer Network guidelines [2].

The criterion for diagnosing lung cancer is a pathologist's diagnosis of biopsy tissue. On the other hand, diagnostic precision is less than 80% [3]. The four most prevalent malignant lung tumor subtypes are squamous carcinoma, adenocarcinoma, small-cell carcinoma, and undifferentiated carcinoma [4]. To make the optimal treatment decisions, scientists must employ the proper techniques to diagnose distinct cancer subtypes during the biopsy. After the National Lung Screening Trial (NLCT), the leading cancer research and training organization, developed a method to use a low-dose helical computed tomography (CT) to detect lung cancer nationwide in 2015, scientists were finally able to use low-dose CT to diagnose lung cancer nationwide. Furthermore, the Dutch-Belgian lung cancer screening trial, the world's second-largest randomized control trial, confirms the advantages of lung cancer screening [5]. However, implementing the US and prospective lung cancer screening in Europe would likely lead to many whole-slide histopathology images, biopsies, and excised tumors. Researchers have proposed many medical image analysis methods in CT scans to segregate the lung parenchyma region automatically [6]. For example, authors in [7] describe signal thresholding strategies based on contrast information for most methods. Because of their lower densities than the rest of the body, the lung region looks darker when framed by a denser region. The underlying framework of these approaches is straightforward and effective for normal lung segmentation. Still, they fall short when expanding the word “lung” to include aberrant tissues, blood arteries, and normal lung tissues [8]. First, it is crucial to obtain a segmented region using iterative thresholding and then refine the obtained region using an opening-closing morphological operator. Significant success has been found in noninvasive therapy and clinical examination in the health industry, especially when utilizing medical image analysis [9]. Researchers use CT imaging for specific diagnostics, and hence, images such as X-rays, MRIs, and CTs are effective therapeutic methods. Because cancer is the deadliest disease, the value of CT images grows even further, given that 1.61 million individuals die from lung cancer each year, according to the World Health Organization [10]. Despite the progress made in medical imaging technology, including CT scans, lung cancer accounted for 76 million deaths in 2018, and about 13% of those newly diagnosed with lung cancer die from cancer [11]. Most cancer deaths occur in low- and middle-income nations, as over 70% of cancers are found in these regions [12]. The automated identification of lesions and automatic categorization of lung diseases have seen significant advancements in CT scans during the last two decades [13]. Machine learning (ML) systems have played a key role in processing images.

Recently, there has been a significant increase in the attention paid to deep learning (DL) in several domains, including image recognition and biomedical image analysis [14]. After retrieving CT scan features, image processing techniques are applied to the image data to assess whether the patient's cancer is benign or malignant.  Figure 1(a) displays a lung cancer nodule view, and Figure 1(b) shows an arrow that indicates a 1.25 mm thick CT slice.

As seen in Figure 1, smaller nodules are in almost any CT scan indicative of problems. For example, the arrow on Figure 1 (b) indicates a tiny nodule to be malignant.  Table 1 displays the causes and detection phases of lung cancer.

The objectives and justification of the work are as the following:

This study was aimed at developing a DL-based automated lung cancer tumor segmentation network utilizing CT scans.

- In current procedures, the lung images were taken and subjected to segmentation, to benefit from the support vector machine classifier [16]
- The present framework has a restriction as it could not predict the type, form, or size of the tumor, and it dealt with several pixels, which is not beneficial for the early detection of cancer. Now, when artificial neural network (ANN) develops a testing solution, it does not reveal some information as to why and how. This diminishes trust in the network
- Neural networks (NN) are a black box and have been confined in their capacity to perceive the potential causal links expressively. On the other hand, NN features deep networks with numerous hidden layers and is helpful for modeling complex systems. However, the training process is again more complex and constantly sensitive, creating a few complications
- It is expected that by applying this model, many current data mining and image processing procedures operate jointly in numerous ways. However, the fundamental drawback of the linear discriminant analysis approach is that it only differentiates the images having abnormalities
- Because of the issues with classifiers, segmentation performs better in accuracy

The contribution of this work is as below:

- This research presents a lung segmentation utilizing 3 traditional and a novel model. This study was aimed at developing a DL-based automated lung cancer tumor segmentation network utilizing CT scans
- Developed a methodology, SegChaNet, that achieves the state-of-the-art performance on numerous segmentation tasks dealing with lung cancer segmentation; of foremost importance is the increase acquired in the precision of tumor segmentation
- Using the channel attention module (CAM) to achieve the goal of managing the feature selection of the bottom-level feature map
- Consequently, this study reveals the capability of early detection of lung cancer, which is known to improve treatment outcomes

The rest of the paper is structured in the following way. The next section contains several examples from the literature and will contrast them with the present study. Next, we explain the methods in Section 3, including methods for the segmentation of lung cancer. Then, we have presented a detailed analysis of the proposed model in Section 4. In addition, the results and a discussion are in this section. Finally, we summarize the full text in Section 5 and present the future work.

## 2. Literature Scan

Numerous studies on lung segmentation have been conducted using conventional image processing techniques such as thresholding, edge detection, and clustering [17, 18]. When faced with chaotic input images, many image processing algorithms resort to primitive techniques and perform poorly. This project was aimed at developing an automated lung cancer tumor segmentation network based on deep learning using CT images. Researchers are examining lung segmentation using convolutional neural networks (CNNs). The researchers now want to enhance lung segmentation performance through complex image segmentation network topologies and other strategies such as attention modules. It has been demonstrated that the attention mechanism significantly improves performance on many DL-based activities.

As a result, our research focuses on segmentation techniques based on attention. For example, attention U-Net [19] outperforms U-Net by sandwiching an attention module with a fundamental structure between the current U-Net structure's contracting and growing channels. Similarly, the authors of [20–22] enhanced the structure of the corrective adversarial network, which was the first attempt to use adversarial learning for lung segmentation on chest X-rays by incorporating attention U-Net and focal Tversky loss for the generating network and binary cross-entropy, respectively.

Additionally, the researchers in [23, 24] used CC-Net as the backbone network, an image segmentation network based on the criss-cross attention module. Additional learning data were generated using image-to-image translation. XLSor is state-of-the-art software. This project was aimed at developing an automated lung cancer tumor segmentation network based on deep learning using CT images. Numerous lung image segmentation networks use a reference lung segmentation model based on chest X-ray images [25].

In their study, the authors in [26] proposed an algorithm for classifying lung nodules by considering the data learned from tissue, shape, and the D technique. This algorithm utilized a “gray level coformation matrix”-based surface identifier, a Fourier shape identifier, and CNNs to train the properties of nodes to depict the heterogeneity of nodules. However, the authors in [27] focused on computer-aided diagnosis (CAD), which they designed manually, so it is not ideal or sufficient for the solution.

U-Net employs the skip connection, which is symmetrical, to directly supervise and lose back propagate on semantic features instead of using these other procedures. The aspect of scale integration permits the implementation of various features from multiple sizes to support multiscale prediction. Because of this, U-Net is primarily used in the medical imaging industry [28]. The researchers in [29] suggested using a recurrent; the residual convolutional neural network (RRCNN) was introduced in conjunction with a U-Net to train more complex networks and extract deep semantic information. The results obtained using R2U-Net in the vascular, lung, and skin datasets are above expectations. As a result, the depth of the U-Net network varies according to the applications it serves. As a result, Liang et al. designed U-Net, which included smaller-scale U-Net levels in larger-scale U-Net levels, with deep supervision, which allows the network to self-select the appropriate amount of depth via training [30].

On the other hand, the researchers in [31] developed the cellular neural network algorithm to detect lung cancer symptoms. In this study, the authors employed X-ray images and thus the CNN algorithm to diagnose lung cancer. The authors in [32] focused on developing CNNs for lung cancer screening in CT scans. The researchers in [33] used multilayered neurons with independent principal components to diagnose lung cancer.

In their study, the researchers in [34] performed a diagnostic classification of lung nodules using 3D-CNNs. They did not foresee overfitting in their model, so they had to include a retraining phase method to address issues linked to image label imbalance. Chon et al. [35] proposed a method that uses an ANN community chart to differentiate benign from cancerous lung nodules. The experimental results show that the scheme has 78.7% classification accuracy [36]. On the other hand, the authors in [37] utilized an ANN model with a classification accuracy of 92 percent in their study. Zhang et al. [38] presented a methodology with an accuracy rate of 75.01% using the Automatic coder (AC), a DL technique.  Table 2 includes the comparison of the literature review in the related field.

## 3. Methodology

### 3.1. Data Acquisition

Images of 46,698 CT scans, both with and without tumors, from the Cancer Imaging Archive (https://wiki.cancerimagingarchive.net/display/Public/RIDER+Lung+CT) were made available. 80% of the data were used for training and 10% for validation to obtain a reliable and accurate network, while the remaining 10% of the data were for testing. We have used different parameters for training segmentation models. We have applied the data augmentation steps to the data. On each patient's scan, we employed intensity normalization based on the mean and standard deviation of the intensities. We implemented our models on a machine with an NVIDIA GeForce RTX 2080 8 GB and Intel Core i9-9980hk processor configuration. We utilized Python (3.8.12), the major programming language, for constructing the framework's subsequent phases. The proposed architecture is implemented using the libraries Anaconda3 (64-bit), Jupyter Notebook, TensorFlow, and Keras.

As seen in Table 3, the dataset is split into train, test, and validation. The CT scan slices are as with tumors and without tumors.

### 3.2. Preprocessing CT Scans

Preprocessing CT scans dealing with high variation in data is a typical job performed during preprocessing. The first step was to truncate all the Hounsfield unit (HU) values between −1000 and 400 [52]. The HU is a metric that measures the density of materials where the air has a value of −1000 HU and bone has a value of 1000 HU; values outside the range of −1000–400 is not considered necessary for lobar segmentation [18]. We then normalized the CT scans to a zero mean with unit variance. To fit the images into a 3D model, we resized all the images and made them the same size, satisfying the memory constraints of the GPU. Two main approaches to this task achieve similar performance: downsampling CT images or applying a patch-based method by partitioning the images into overlapping patches. Since we needed to incorporate tracheal and bronchial segmentation as an auxiliary task into the segmentation, we opted for the downsampling technique, ensuring that the trachea and bronchi were present in each image. The size should be the same on all three axes to downsample the image [53]. If one axis is of better resolution than another, the performance along lower resolution axes is worse, as they contain less information than the other axes. All the CT scans, with their masks, were resized to 128 × 128 × 128 using linear and neighbor interpolation, respectively, as it was the most significant cube size shape we could fit into memory. What makes SegChaNet different from U-Net is that U-Net was initially designed for medical image interpretation and segmentation, while we developed SegChaNet for lung image segmentation.

U-Net has a wide variety of industrial applications and has played an important part in the development of the image automation society. The architecture of SegChaNet is defined by its appealing and expansive components. The contracting path comprises several convolutional patches with 3 × 3 filters and unity strides in both directions, which are preceded by ReLU layers. This path takes the input and extracts the key features, yielding a feature vector of a certain length. The second path uses information from the contractive path to creating an output segmentation map by copying and cropping the feature vector using upconvolutions. The exploit that connects the first and second channels is vital for this system. This connection enables the network to get very precise information from the contractive route, developing a segmentation mask close to the desired output. SegChaNet benefits from extremely asymmetric datasets because of its composition of big chunks of lung images. Due to the lungs' different geometries and image density distributions, it is difficult to distinguish them in clinical ultrasound images automatically.

SegChaNet resembles U-Net but as explained above, combining two different paths, and utilizing Binary cross Entropy, integrated with the Channel Attention Module, differs it from the rest. The encoder layers are similar to the convolutional layers of the U-Net.

For SegChaNet, nine distinct hyperparameters are used in training to determine the optimal configuration. These training hyperparameters are listed in Table 4. For training purposes, all trials were done in 500 epochs for training purposes. Training time variation was small across networks, with an average of 18 minutes.

### 3.3. U-Net Model

U-Net is a technique for automatically segmenting images. U-Net is a pixel-based image segmentation algorithm for various architectural and convolutional neural network layers. It outperforms traditional models in terms of success. It also performed well on datasets with a minimal number of photos. The term “U-Net” comes from its U-shaped design. U-Net is made up of encoding and decoding components. The content of the images is recorded in the code section. It is made up of top pooling layers. On the other hand, the decoding portion is the symmetric expansion route utilized to obtain exact localization via the use of delegated convolutions. The U-Net model is shown in Figure 2. Each of the 32 × 128 × 128 voxels included inside the input layer corresponds to a single channel. We did 1D convolution on the input by applying a 1 × 3 × 3, 2 × 3 × 3, and 1 × 1 × 1 filter. Using max pooling, we perform one-dimensional max pooling. By using 1D upsampling, the voxel size was raised from 2 2 to 4 4. To model U-Nets, we use the rectified linear unit (ReLU) as the input and the sigmoid function as the output layer's activation function. Data augmentation is a strategy that may assist avoid overfitting and increase performance by increasing the quantity of data points. The left-to-right inversion and white-to-black inversion methods were used in this work to provide data augmentation. We used Adam as an optimizer because of its adaptive moment estimation. To arrive at the ideal learning rate, various values were tried, including those between 0.3 and 0.1, with every successive change made along with the range. To optimize a solution, we must minimize the loss function, the difference between the projected result, and the correct answer. We calculated these equations to get the following:

(1) $$\begin{array}{c} \begin{array}{c} \text{Loss function}=2-\left\{\text{IOU}\left(A,B\right)+\text{DSC}\left(A,B\right)\right\},\\ \text{IOU}\left(A,B\right)=\frac{\left|A\cap B\right|}{\left|A\cup B\right|},\\ DSC\left(A,B\right)=\frac{2\left|A\cap B\right|}{\left|A\right|+\left|B\right|}. \end{array} \end{array}$$

In this case, the estimated value, *B*, is an estimation and the actual value, *A*, is accurate. The intersection over union (IOU) and dice similarity coefficient (DSC) are represented as the Jaccard Index (JI). The JI and the DSC are both methods of measuring class similarity. To determine the accuracy of contour demarcation, we use DSC. The ensemble learning for five inference results comprises 5-fold cross-validation; afterward, we obtained DSC for U-Net. The following example illustrates this principle in ensemble learning, for which we have found a pixel value of 1 for three inferences but a value of zero for two inferences. In this case, we selected a majority value of 1.

In Figure 2, the path has two distinctive sections: a contracting section and an expansive one. A typical convolutional architecture often features a contracting path. It is a 2 × 2 max pooling with stride 2 and a ReLU followed by two unpadded convolutions such as 3 × 3 convolutions. We have increased the amount of feature channels by a factor of two each time while performing downsampling. The enlarging path has upsampling, followed by 2 × 2 convolutions.

### 3.4. V-Net Model

We applied the V-Net architecture using the TensorFlow and Keras frameworks in Anaconda, as stated in Data Acquisition. We have employed the V-Net, an autoencoder, for 3D image segmentation. Its residual connections aid networks to converge and perform well on small datasets.  Figure 3 shows the model's architecture, where the input image is 128 × 128 × 128 × 1 (height, width, depth, and channels) and passes through six encoder layers. As seen from Figure 3, V-Net, we used convolutional layers with a stride of 2 × 2 × 2 instead of the max pooling operation. The last layer before each output was a 1 × 1 × 1 convolution with a softmax activation function that gives us the probability that each voxel belongs to one of the classes. Various regularization techniques enhanced the model's generalizability, including dropout and batch normalization. Training the model on distinct but relevant tasks has been shown to increase a model's performance. The model's performance is measured using the DSC, a function of sensitivity and specificity typically used in segmentation studies, permitting a comparison of our model's performance to others. We compared our model to other models by researchers who released the original dataset. A *p* value obtained using a *t*-test, more diminutive than 0.05 between the models, was considered statistically significant for independent comparisons.  Figure 3 shows V-Net architecture.

We illustrate our CNN using the schematic in Figure 3. To both find features in the data, we use convolutions, as well as to reduce the resolution after each stage by employing stride suitable to the level. In the left portion of the network, we used a compression path to reduce the file size, and in the right portion, we decompressed the file until we reached its original size. We employed all of the convolutions with the proper amount of padding.

### 3.5. SegChaNet Model

Segmentation tasks generally concentrate on learning multiscale features and the integration of local and global contexts. However, computationally demanding training segmentation networks including these qualities and implementing these directly on volumetric data is difficult. To help promote multiscale learning, we integrate CAM convolutions into the network and place these convolutions at the very end of the feature extraction process. They work together with the output of the decoder layers to promote the learning of multiscale features. We use this connection to assist the training of network gradients as well. We maintained residual links between the decoding component and the alteration when we adjusted. The proposed network consists of four blocks of encoders and decoders each using two 3D convolution layers with a 3 × 3 × 3 kernel size and a batch normalization and leaky ReLU activation function.

However similar it may seem, SegChaNet varies from U-Net. For example, we use the maximum linked component detection to extract the whole region, and SegChaNet additionally takes use of CAM. Besides, preprocessing steps have been applied before the SegChaNet model is applied. So, it necessarily comprises a preprocessing phase.  Figure 4 displays the main novel architecture.

As seen in Figure 4, this decoder uses a 2× upsampling method. We proposed the convolution of the augmentation module's CAM convolution layers such that the first layer utilizes a dilation rate of one, and each subsequent layer doubles the dilation rate. It is upsampled to scale each decoder's output, followed by all concatenated outputs.

#### 3.5.1. Channel Attention Module

This section delves further into SegChaNet's model architecture (illustrated in Figure 4). Because of its higher performance, the pixel-level classification strategy is employed in medical image segmentation tasks based on the U-Net model. We included the cross-level feature fusion module (CFFM) in our end-to-end network architecture, SegChaNet, to create a merged network with two primary components and CAM. The CFFM enables the fusion of features from the top-level feature map into the feature map of the bottom layer, allowing the CAM to regulate feature selection in the bottom-level feature map. The second component is the U-Net, a two-part encoder-decoder architecture in which the first half is used to extract features and the second half is upsampled. Special caution is required when using a skip connection topology between the encoder and the decoder. Additionally, a skip link was used to connect the downsampled and upsampled feature maps. The CAM and architecture used are shown in Figure 4. Because the high level includes much semantic information, it may help guide the low-level choices. Several studies have shown that attentiveness is vital in human perception. Recently, attention processes have been included in complicated sequences and transformation models for various activities. Channel attention modules, in particular, have been utilized to boost deep learning performance in a variety of computer vision applications. DL methods for image classification and semantic segmentation rely on continuous fundamental convolutional processes. Consequently, deep learning networks can only manage the local components of an image, resulting in the loss of global information.

A sophisticated method must be used to estimate the parameters. The parameters of the investigation were determined in three steps. Attenuation coefficients can be derived from the attenuation profile using a single-path model and a least squares estimator. The number, position, and amplitude of key pathways may be calculated from the impulse response using a basic peak detection approach. In simpler cases, this phase usually gives enough precision. To expand the number of pathways, parameters must be developed using either impulse response or amplitude and phase responses. To estimate parameters, complex procedures must be applied. The parameters of the investigation were determined in three steps. An initial estimate of the attenuation coefficients can be generated from the attenuation profile using least squares estimators. The number, position, and amplitude of key pathways may be calculated from the impulse response using a basic peak detection approach. In most cases, this is all that is required. To increase the number of pathways, the parameters must be further changed through an evolutionary process employing quality criteria such as impulse response or amplitude and phase response.

We have provided a more specific resolution information option. Furthermore, the SegChaNet model may learn the weight of each channel via CAM, resulting in attention in the channel domain. The CAM procedure is as follows:

(2) $$\begin{array}{c} X_{\text{cam}}=\text{CAM}\left(X_{L},X_{H}\right), \end{array}$$

where *X*_cam_represents the output of the CAM module and *X*_*L*_ and *X*_*H*_ represent the low-level feature map and high-level feature map, respectively.

(3) $$\begin{array}{c} x_{\text{cam}}^{i,j,k}=x_{gL}^{i,j,k}+\text{up}\left(x_{H}^{i,j,k}\right), \end{array}$$

where *x*_cam_^*i*,*j*,*k*^ represents the pixel value of the *i*th row, *j*th column, and kth channel in the output feature map of the CAM.

In addition, *x*_*H*_^*i*,*j*,*k*^ H is the pixel value of the *i*th row, *j*th column, and *k*th channel of the high-level feature map. up (.) means the bilinear interpolation.

(4) $$\begin{array}{c} X_{gL}=\text{Conv}1\left({\left[X_{L}^{\prime k}\times g\left(X_{H}^{k}\right)\right]}_{k=0}^{k=c-1}\right). \end{array}$$

Global pooling transforms the feature map *X*_*gL*_ and low-level feature map *X*_*L*_. The 3 × 3 convolution operation adjusts the feature map size and merges the channel features. Still, because the low-level and high-level features' feature map size and channel number are different, the low-level feature needs a 3 × 3 convolution operation.

(5) $$\begin{array}{c} X_{L}^{\prime }=\text{Conv}3\left(X_{L}\right). \end{array}$$

Global pooling, convolution with a 3 × 3 convolution kernel, and convolution with a 1 × 1 convolution kernel which are known as *g*(.), conv3(.), and conv1(.), respectively. The letter “c” denotes the total number of channels [54].

When global pooling is used, CAM gives an initial global context that serves as a guide for recognizing low-level features. To decrease the number of feature mappings in the encoder, we first apply three convolution filters to the low-level features. A global context is created by multiplying the low-level features by the high-level features using a 1 × 1 convolution process. Finally, we have combined low-level and high-level features. Thus, the CAM module uses scale feature maps more effectively while delivering information to lower-level feature maps.

When it comes to the model's performance, as seen, Table 5 shows the performance of the U-Net method with and without CAM.

As seen in Table 5, accuracy of the U-Net method without CAM is 88.61.21 while with CAM is 95.94.  Table 6 displays the methods and performance of the V-Net method with and without CAM.

From Table 6, the accuracy of the V-Net method without CAM is 87.35 while with CAM is 95.75.  Table 7 shows the methods and performance of the novel method SegChaNet with and without CAM.

From Table 7, it is evident that the accuracy of the SegChaNet method without CAM is 96.81% while with CAM is 98.48.  Figure 5 shows the performance of SegChaNet, illustrating the comparison of the novel model with the state-of-art ROC performance.  Table 8 compares models' accuracy evaluated in DSC, JI.

Table 8 displays the results with CAM. As seen, SegChaNet is far better when compared with the other methods.

From Figure 5, it is evident that the AUC of V-Net, U-Net, and SegChaNet without CAM is lower when compared with used models plus CAM.

### 3.6. Training Procedures

We are creating a new model from scratch and will use the DSC, JI, and normalized surface distance to test it. We computed normalized surface distance as a combination of the model-predicted segmentations that overlap with the ground truth. In the segmentation process, we utilized these variables to determine segmentation accuracy. Segmentation networks' segmentation binary cross-entropy is commonly employed. As proposed, we employed binary cross-entropy and DSC loss functions to train the networks in this investigation. The loss value applied on SegChaNet is in Equation (2), proving that the overall loss is less sensitive to class imbalance. Our tests found greater segmentation accuracy when utilizing the binary cross-entropy over the individual loss. The equation in [55] is as follows:

(6) $$\begin{array}{c} \zeta \left(y,\hat{y}\right)=\zeta_{dc}\left(y,\hat{y}\right)+\zeta_{bce}\left(y,\hat{y}\right). \end{array}$$

In Equation (6), $\hat{y}$ denotes the model's output, and the ground truth labels are denoted by *y*. We use the two-class version of the DSC loss $\zeta \left(y,\hat{y}\right)$ proposed in [56], a fully connected DL model trained on 500 epochs with an Adam optimization learning rate of 0.0005. If the validation binary cross-entropy did not improve after 15 epochs, we would reduce the learning rate by 0.1 per ten epochs. We updated the dataset with additional random rotations and flipping to help minimize overfitting and improve the resilience of our technique to varied hippocampus shapes. Our research noticed that the segmentation masks became poorer during additional large rotation angles. So, to remain consistent, we reduced the rotation angles to fall within roughly 10 degrees.

### 3.7. Evaluation Metrics

The precision of segmentation directly affects the success or failure of the segmentation process. Therefore, three measurement variables, DSC, sensitivity, and specificity, are utilized to assess the accuracy of the suggested techniques. In addition, true positives (TP), false positives (FP), true negatives (TN), and false negatives (FN) are also crucial in the assessment [57].

Dice: designed to evaluate the overlap rate of prediction results and ground truth. DSC ranges from 0 to 1, and the better-predicted result will have a more considerable DSC value.

(7) $$\begin{array}{c} \text{DSC}=\frac{2\text{TP}}{2\text{TP}+\text{FP}+\text{FN}}. \end{array}$$

Sensitivity (also known as the true positive rate or the recall) indicates the percentage of genuine positives that are accurately detected.

(8) $$\begin{array}{c} \text{Sensitivity}=\frac{\text{TP}}{\text{TP}+\text{FN}}. \end{array}$$

Specificity (also called the true negative rate) measures the proportion of correctly identified actual negatives.

(9) $$\begin{array}{c} \text{Specificity}=\frac{\text{TN}}{\text{TN}+\text{FP}}, \end{array}$$

where TP denotes the true positive voxels, TN denotes the true negative voxels, FP denotes the false positive voxels, and FN denotes the false negative voxels. We use the 4-union (IOU), DSC value, and Hausdorff distance [58]. Here, we defined IOU as

(10) $$\begin{array}{c} \text{IOU}=\frac{\text{TP}}{\text{FN}+\text{FP}+\text{TP}} \end{array}$$

To understand what this output means, think of a medical test proposed target capture, in which a group of clinicians manually label the target region, and the network prediction shows the areas around it.

The intersection and union of two sets are equivalent when defined as the IOU ratio [59]. Researchers use the IOU score widely to quantify pixel-level image segmentation performance in image recognition algorithms. IOU can have a value from 0 to 1. As the IOU increases, the overlap between the two zones will decrease and vice versa.

## 4. Results and Discussion

As demonstrated in Figures 2 and 3, we enhanced lung cancer segmentation in the proposed model SegChaNet by comparing it to two state-of-the-art models. Despite having almost identical encoder and decoder designs, U-Net structures and their variants outperform non-U-Net structures. While decoders on other networks employ the addition operation, the skip connector and upsampling set of inputs are concatenated in the decoder. We lowered the data dimension to compensate for the value lost during the addition procedure. In addition, to impact the behavior of other network features, we paired SegChaNet's encoder and decoder with a large number of recurrent, residual convolutions. As a result, when we utilized SegChaNet to evaluate the CT scan dataset, we found that it was prone to overfitting. That is why we used CAM, which performs a function by correctly utilizing all of the feature information on each level. Unlike attention U-Net, which segments the esophagus with an air hole, the SegChaNet considers the air hole a boundary when segmenting. Furthermore, U-Net cannot identify small airways [60], required for esophageal analysis. This is due to the underutilization of complex features. However, neither can they use the features of several layers to guide feature selection, nor can they combine low-level and high-level features with driving feature selection at a lower level. On the other hand, CAM uses the channel to combine the features of many stages.

In contrast, CFFM selects low-level, fine-grained features based on high-level semantic features, resulting in the network producing features on the shape and border of the esophagus. As a result, we achieved our primary goal of enhancing segmentation effects and generalization capacities.  Figure 6 depicts a comparison of the DSC coefficient performance of the employed models.

When compared to other works in the literature, such as segmentation techniques in [61], we can observe that, while they have profited from alpha attribute maximization, the result is not as expected, with an IOU of 74.18 percent and 84.80 percent. Furthermore, compared to 3D-U-Net neural in [62], they used 3D U-Net, and their DSC performance reached 95.30 percent. Speaking of which, the SegChaNet approach performs significantly better.

As seen from Figure 6, V-Net shows a good performance, but it fails in the final part, while the best performance is from the SegChaNet model. For the first 20 epochs, U-Net shows the worst performance.  Figure 7 displays marked images using grad cam.

As seen in Figure 7, we have marked images using grad cam. Also, we utilized the DSC, JI, and normalized surface distance (NSD) with 4 mm performance to test various networks. As illustrated in Figure 8, we examined the segmentation performance of V-Net, U-Net, and U-Net and V-Net with CAM convolutions. The V-Net attained mean DSC scores of 95.75% without CAM, 87.35% for the training, validation, and test sets. At the same time, the U-Net results match the V-Net scores relatively well. CAM convolutions allowed U-Net to improve the scores to 88.61% and 95.94%. The proposed technique demonstrated 96.81% without CAM and 98.48% with CAM for the training, validation, and test sets.

Furthermore, our method outperformed other cutting-edge networks for both the JI and NSD metrics. This is highlighted clearly.  Figure 7 shows the segmentation quality of the proposed method next to other methods so that it can be compared visually. When used to color coordinate ground truth with predictions, red represents the ground truth, while yellow, green, and cyan represent the V-Net, U-Net, and method provided in this article predictions. The top-right area of the mask in Figure 7 comprises small discontinuous portions; we demonstrated the advantage of CAM convolutions by effectively segmenting such small sections. However, when the learned qualities become more prevalent worldwide, the U-Net and the suggested method might effectively gather the regions. Figure 8 depicts the three-dimensional surface meshes of two different patients. We can observe how the SegChaNet model influences our conclusions in the method provided in columns 3 and 4. The bottom boundary of the red component of the hippocampus is about one hundred millimeters below the ground's surface. Figure 8 depicts SegChaNet's top and worst performance ratings.

Figure 8 displays the SegChaNet model's best and worst performance. As seen, the best score is about 95 while the worst one is 51.47.

For the segmentation of lung nodules using low-dose CT imaging, we investigated the imaging features of lung nodules ranging in size from 5 to 32 mm in diameter in cancer patients undergoing low and normal voltage CT scans. This study was aimed at developing a DL-based automated lung cancer tumor segmentation network utilizing CT scan segmentation approaches combined with the assessment of segmentation uncertainty. Additionally, we investigated the influence of two widely used cost functions, dice and JI, on the model output's uncertainty measures. All three segmentation models perform well on the segmentation challenge, with dice-trained models marginally outperforming JI-trained models. The most precise methods for predicting nodule volumes were not the most repeatable, emphasizing the need to evaluate their precision and accuracy. Significant variations in algorithm performance were seen, especially in a sample of heterogeneous nodules, highlighting the need to use the same software throughout a longitudinal study.

In contrast to some recently proposed methods, we aimed to increase segmentation prediction variability by producing segmentation hypotheses with our novel method. Importantly, SegChaNet encompasses the entire space of possible segmentations rather than providing information about the models' uncertainty [63]. As is well known, manual, automated, and semiautomatic segmentation pose difficulties in terms of repeatability. The ability to accurately and consistently target lung cancer regions from surrounding tissues using CT images is critical for the clinical assessment of disease progression. The obtained features contribute to SegChaNet throughput and are subsequently decoded to provide an automatic network segmentation. In addition, these features are expected to encapsulate some of the intratumorally and peritumoral area's complex structural and functional geometry, some of which may be related to cancer survival. Overall, we show that SegChaNet, when combined with UQ, shows the best accuracy in lung cancer segmentation. When the existing V-Net models' results are studied, a novel SegChaNet model is proposed that capitalizes on the SegChaNet's superior qualities over the V-Net and U-Net models. On this dataset, three models were run, including the SegChaNet model, and the organ and tumor segmentation procedures were carried out independently. It has been shown that V-Net models can efficiently segregate organs and tumors using computerized images and that by handling the coding and decoding phases separately, more successful models may be developed than present V-Net models. Using medical imaging may be possible to develop more accurate models for multiorgan segmentation. The study may potentially be utilized as a reference for future SegChaNet models due to the success of the original SegChaNet model implementation and the beneficial contribution of the CAM architecture. Since the CAM design was applied solely to the output layer, tiny segmentation characteristics may be recorded. This is crucial for model design since each parameter is only effective when introduced to the appropriate model blocks.  Table 9 compares the SegChaNet segmentation model's performance to that of other leading-edge studies.

Table 9 shows the performance of the SegChaNet segmentation model compared with other state-of-the-art works. Because of utilizing preprocessing stages and UQ methods, SegChaNet demonstrates the highest accuracy and dice outcomes.

## 5. Conclusions

The primary goal of this work is to offer a practical approach to lung segmentation. This paper describes a novel method, SegChaNet, that compared two traditional models (V-Net and U-Net) for lung cancer segmentation in CT scan images. SegChaNet achieves its top performance by utilizing a U-Net framework with CAM convolutions in the network's deepest layer and substantial supervision in its decoder layer. The proposed architecture surpasses state-of-the-art methods in segmentation accuracy and demonstrates initial feasibility in autosegmentation of the lung. Furthermore, it is likely to perform with various datasets and apply to other segmentation challenges in medical imaging. Overall, the SegChaNet method without CAM is 96.81% while with CAM is 98.48%.

Future studies will focus on whether the segmentation results help clinicians in the clinical setting while treating cancer. Additionally, we believe SegChaNet still has potential for improvement in terms of computing costs.

## Figures and Tables

**Figure 1:** (a) Lung cancer nodule view. (b) An arrow indicates this 1.25 mm thick CT slice to contain approximately 2 mm long lung nodules.

**Figure 2:** U-Net architecture.

**Figure 3:** V-Net architecture.

**Figure 4:** An encoder-stage-to-decoder stage residual connection network architecture. The encoder uses residual connections and 3D max pooling operations.

**Figure 5:** SegChaNet, U-Net, and V-Net model with and without CAM.

**Figure 6:** Applied model dice coefficient.

**Figure 7:** Marked images using grad cam.

**Figure 8:** SegChaNet's best and worst performance scores.

**Table 1:** Lung cancer: causes and prevention.

(i) Detection of lung cancer is generally difficult because specialists cannot find the infected area until it reaches the next stage. As a result, the chance of survival for lung cancer, in 54% of detected cancers, not in the advanced stages, with early intervention, is only 4% [15].

(ii) The probability of increasing lung cancer diagnoses due to the number of cigarettes consumed and sometimes after drinking is proportional. As a result of harmful habits, a minor case of lung cancer may occur even in individuals without disease risk.

(iii) X-ray, CT, or MRI scans are performed to examine lung cancer and differentiate abnormal lung development. The best technique is CT, which experts can overlook when not in ML.

**Table 2:** Comparison to the literature works.

References	Datasets	Method	Result (%)
Chaturvedi et al. 2019 [39]	LUNA 16	3D DL DÖ, V-Net architecture	Sensitivity: 96.5 FP:19.7
Chapaliuk et al., 2019 [40]	ACDC LUNGH	VGG16, ResNet50, and CNN	Sensitivity: 97.9 Accuracy: 93
Petrellis et al., 2018 [41]	UCI	Gaussian blur, Otsu thresholding	Sensitivity: 87 Accuracy: 97
Yuan et al., 2019 [42]	134 BT Shandong hospital	Watershed transform	Sensitivity: 88.8 Accuracy: 90
Cao et al., 2016 [43]	LUNA16	3D and 2D CNN	Precision: 87 Sensitivity: 99.1
Xie et al., 2019 [44]	LUNA16	2D CNN and RCNN	AUC: 95.4
Sun et al., 2017 [45]	LIDC-IDRI	CNN, deep belief network, and Boltzmann machine	Sensitivity: 82.2 AUC: 81.8
Huang et al., 2018 [46]	LIDC-IDRI	CNN, extreme learning machine, and deep transfer	Sensitivity: 91.6 Accuracy: 86.5
Pehrson et al. (2021) [47]	LIDC-IDRI	This study was aimed at developing a DL-based automated lung cancer tumor segmentation network utilizing CT scans	Sensitivity: 91.7 Accuracy: 93.8
Sharma et al., 2011 [48]	LIDC-IDRI	Diagnostic indicators	Accuracy: 80.1
Akram et al., 2012 [49]	LIDC-IDRI	Neurofuzzy	Accuracy: 95.5
Paulin et al. 2011 [50]	LIDC-IDRI	For MLP SVM training, the back propagation technique is employed	Accuracy: 83.6
JIA et al. 2007 [51]	NCA	For MLP SVM training, the back propagation technique is employed	Accuracy: 92.4

**Table 3:** Some distinct sorts of CT scan slices in the dataset.

Data		Number of patients	Tumor	Without tumor	Notes
Train		370	14,848	20,840	35,688
Test		90	4520	4740	9260
Validation		50	850	900	1750
Total		510	20,218	26,480	46,698

**Table 4:** Hyperparameters used for training SegChaNet.

Exp.	SegChaNet	
	ILR	Minibatch
1	1e−4	2
2	1e−4	8
3	1e−4	12
4	1e−3	2
5	1e−3	4
6	1e−3	8
7	3e−3	4
8	3e−3	12
9	3e−3	8

**Table 5:** U-Net method with/out CAM performance.

U-Net method	Dice (%)	Sensitivity	Specificity	Precision	*F*-measure	Accuracy (%)
Without CAM	88.61	97.45	93.12	93.01	93.21	93.21
With CAM	95.94	97.62	90.43	89.87	95.56	95.14

**Table 6:** The V-Net method with/out CAM performance.

V-Net method	Dice (%)	Sensitivity	Specificity	Precision	*F*-measure	Accuracy (%)
Without CAM	87.35	88.29	84.74	86.51	91.14	91.63
With CAM	95.75	96.96	89.77	89.21	94.91	94.48

**Table 7:** SegChaNet method with/out CAM performance.

SegChaNet	Dice (%)	Sensitivity	Specificity	Precision	*F*-measure	Accuracy (%)
Without CAM	96.81	93.79	90.19	92.15	96.89	96.47
With CAM	98.48	92.82	94.08	96.66	98.49	98.90

**Table 8:** Evaluation of segmentation accuracy in DSC, JI for 3 models.

	Training	Val	Testing	
Models	DSC	DSC	DSC	JI
V-Net	0.953	0.907	0.893	0.949
U-Net	0.955	0.893	0.911	0.956
SegChaNet	0.989	0.947	0.937	0.957

**Table 9:** Comparison of the performance of the SegChaNet segmentation model with other state-of-the-art works.

Author (year) [reference]	Dataset	Accuracy	Qualitative analysis	Conclusion
Skourt, BA, et al. (2018)	MV, MI, and ME (union) auto: MV phase	0.95	The number of patients with nDSC 1 (within 1-millimeter uncertainty): 7. There are no discernible differences between b-spline and demons	With autocontouring, one may get sharp edges and corners.

Wouter R. P. H., et al. (2021)	All processes are done manually. Auto: dependent on the amount of artifacts, either ME or MI	0.76	NA	In the main breathing phase, there is good agreement between ITV and GTV with manual contours.

Mingjie X., et al. (2019)	Manuel: every stage auto: inherited from the MI phase	0.95	The number of patients that need manual adjustment	Good agreement between auto and manual contours.

Xu, M, et al. (2019)	Manual: all phases Auto: propagate from MI phase	0.92	Minimal. NA	Although autocontouring is precise, it produces bigger shapes.

Qinhua, H., et al. (2020)	Manual: every stage auto: propagated from ME phase	0.94	NA	Deformed contours agree well with physician-drawn contours.

Chiu, T. W., et al. (2021)	Manual: every stage auto: propagated from ME phase	0.63	The propagated IGTVs were mostly within the mIGTVs	The rigid body propagation method generates ITV within a 1 mm margin of error.

Jiang, J. et al. (2018)	Manual: ME (expert) and MI phase auto: ME phase	0.74	NA	The algorithm utilized generated more precise results. Results of segmentation differ from those in previously published papers.

SegChaNet (the proposed network)	Images of 46,698 CT scans both with and without tumors from the cancer imaging archive auto: ME phase	98.90	The applied preprocessing steps	A combined network with two primary components with many CAM has been utilized. We do not employ any manual contours.

## Data Availability

Data sharing is not applicable to this article as no datasets were generated during the current study.
